# Effect Analysis of Clinical Pathway Nursing Combined with Humanized Nursing in Cerebral Infarction

**DOI:** 10.1155/2022/8270137

**Published:** 2022-06-11

**Authors:** Lili Xiao, Tingting Xiao, Fang Yu

**Affiliations:** ^1^Department of Neurology, Ganzhou People's Hospital, Ganzhou 341000, China; ^2^Department of Obstetrics and Gynecology, Ganzhou People's Hospital, Ganzhou 341000, China; ^3^Department of Joint Surgery, Ganzhou People's Hospital, Ganzhou 341000, China

## Abstract

**Objective:**

To make the application effect of clinical pathway nursing combined with humanized nursing clear in cerebral infarction.

**Methods:**

Hundred patients who suffered from cerebral infarction had been hospitalized in our hospital and they become our study objects. By means of the random number table, they were separated into 50 cases both in the control group and in the observation group. The control group accepted the routine nursing, and the observation group accepted the clinical pathway nursing mixed with humanized nursing. The followings were compared including the hospitalization expenses and length of stay, National Institutes of Health Stroke Scale (NIHSS), Barthel index rating scale (BI), Fugl-Meyer Assessment (FMA), and the incidence of complications and recurrence rate. A comparison was made between the two groups about satisfaction with nursing.

**Results:**

In contrast with the control group, the treatment expenses and length of stay in the observation group were considerably reduced (*P* < 0.05). In contrast, before nursing, the NIHSS marks of the two groups decreased considerably after nursing, and the scores of BI and FMA increased considerably, the NIHSS scores of the observation group were considerably lower than those of the control group, and the scores of BI and FMA were considerably higher than those of the control group (*P* < 0.05). In contrast with the control group (44.00%, 12.00%), the incidence of complications (22.00%) and recurrence rate (2.00%) in the observation group were considerably lower (*P* < 0.05). In contrast with the control group (72.00%), the satisfaction of nursing in the observation group (96.00%) was considerably higher (*P* < 0.05).

**Conclusion:**

The application effect of clinical pathway nursing combined with humanized nursing in cerebral infarction is significant. It can not only effectively reduce hospitalization expenses and hospitalization time, improve neurological function, ability of daily living, and limb motor function but also reduce complications and recurrence and improve patients' satisfaction with nursing, which has a high clinical reference value.

## 1. Introduction

Cerebral infarction is caused by atherosclerosis of cerebral artery embolism or directly in a state of occlusion of a disease. Some brain tissues even undergo necrosis and softening due to ischemia and hypoxia, leading to neurological dysfunction [1]. Cerebral infarction occurs frequently in the elderly, which will not only cause significant degeneration of body organs, tissue functions, and physical functions but also cause motor, cognitive, psychological, and emotional disorders of varying degrees [2, 3]. Therefore, certain nursing should be given at the same time as treatment. Conventional nursing is generally limited to the condition of nursing and cannot take into account other aspects of nursing. At the same time, there are also a series of problems, such as weak pertinence, incoherent time, single mode, and inappropriate method [4]. As a standard nursing mode of clinical norms, clinical pathway nursing is a relatively mature operation system, which has been clinically used in the nursing of a variety of diseases and achieved quite significant application effects [5, 6].

Humanized nursing, as a people-oriented nursing mode, is highly consistent with the nursing concept advocated by modern medicine. It runs through the whole nursing process and is a comprehensive, high-quality, and humanized nursing measure, which can effectively improve the quality of clinical nursing [7]. However, there are few research studies on the combined application of clinical pathway nursing and humanized nursing, worth a further research. So, this research chiefly explores the application effect of clinical pathway nursing mixed with humanized nursing in cerebral infarction, aiming to give more information for boosting patients with cerebral infarction clinically life quality.

## 2. Data and Methods

### 2.1. General Information

All 100 patients with cerebral infarction in our hospital from September 2019 to September 2021 were picked as our study objects. By means of the random number table, they were separated into the control group (50 cases) and the observation group (50 cases). The control group accepted the routine nursing, and the observation group accepted the clinical pathway nursing mixed with humanized nursing on its basis. This research was ratified by the hospital ethics cCommittee. There was no obvious distinctions in statistics between the two groups in gender, age, time from onset to treatment, severity of disease, infarct site, and education level (*P* > 0.05), demonstrating comparability; we can consult Table 1.

### 2.2. Inclusion and Exclusion Criteria

Inclusion criteria [8]: ① all patients were determined cerebral infarction by computed tomography (CT) and magnetic resonance imaging (MRI); ② patients without abnormal heart, liver, and kidney function; (3) cognitively and mentally normal patients; (4) patients who are conscious and can communicate normally; ⑤ informed consent was endorsed by patients themselves or their own families.

Exclusion criteria: ① patients who have received relevant care; ② patients with subarachnoid space or parenchymal hemorrhage; ③ patients with brain tumor, epilepsy, intracranial infection, cranial trauma, and other neurological diseases; ④ patients with malignant tumors.

### 2.3. Methods

Control group routine nursing: first of all, explain the pathogenesis of the disease, treatment methods to patients, and their own families. Follow the doctor's advice to use sedatives, analgesics, vasodilators, etc., to implement the treatment of patients, in the treatment process to closely observe the changes of their vital signs. The patients were examined by electrocardiogram to determine the location and degree of cerebral infarction, and the appropriate treatment plan was made on the basis of the actual condition of the patients. Carefully observe the patient's consciousness, urine volume, etc., pay close attention to whether the patient has arrhythmia and other serious complications, once abnormal, and immediately contact the doctor, and then, take corresponding treatment measures. Communicate with the patient and carry on nursing to its psychological condition.

The observation group accepted the clinical pathway nursing combined with humanized nursing ground on the control group. (1) Clinical pathway nursing: management system establishment; the nursing group was established, with the leadership of the head of nursing, and the backbone members included rehabilitation therapists, psychotherapists, medical leaders, and life nurses. The group leader and team members are familiar with and master the implementation method and process of nursing and master the patient access standard and exit standard and variation treatment. Group training is carried out to ensure that members can master the basic contents of nursing. Follow the principles of doctor-patient sharing, multidisciplinary participation, safety, applicability, scientific nature, and so on to formulate nursing programs. The formulation of nursing programs at the same time can also learn from domestic and foreign experience and consult relevant experts, after in-depth discussion to improve the nursing text. Nursing implementation: (1) admission 1∼2 days: first is to introduce the basic hospital environment to patients and their families, assess patient's condition through communication, and participate in patient consultation and rehabilitation assessment. Give health education to patients at the right time and patiently answer questions raised by them. Corresponding health education shall be given according to the specific situation of patients. ② 3∼7 days after admission: maintain active and effective communication with patients and improve patients' understanding of the disease by holding lectures related to rehabilitation. Infection prevention measures should be taken to prevent nosocomial infection. By displaying the mouth shape of speech, the patient can be instructed to exercise the oral and facial muscles, thus laying the foundation for later language training. The patient is told not to be supine position as far as possible and guided the patient to take the affected side, by increasing its perceptual stimulation to lengthen the affected side, reduce spasm. Instruct the patient to extend the upper limbs forward, straighten the elbow, and keep fingers apart and palms up. In the lateral position, the lower limbs were kept upward, ankle dorsiflexion and knee flexion. When taking the seat, keep the trunk straight and ensure the same weight on both hips and the shoulder joint external rotation and forward extension. When changing positions, move slowly and do not move too much. ③ Two weeks after admission: observe the patients' recovery of limb function and guide them to carry out limb rehabilitation training. Guide the patient to train the range of motion of the joint, step by step, according to the order of shoulder, elbow, wrist, finger, hip, knee, and ankle. Each joint was trained 5–10 times, once in the morning and once in the afternoon. When training the shoulder joint, pay attention to the slow lifting of the arm, the head of the refrigerator, and the slow moving. And then slowly move back to your side. When you train your elbow, place your hand flat on your side, straighten your elbow, bend your elbow, and straighten your elbow. In the rotation of the elbow joint, the patient should first hold the palm of the hand so that the palm repeatedly rotates up and down. Wrist joint mainly for internal and external rotation, extension, flexion movement. Knuckle training: hold the patient's wrist, tell him to clench his fist, and then relax the fist; five fingers should be straight. During hip movement, put one hand behind the knee of the patient, raise the leg to 90° as far as possible, and then slowly put the leg back to the original position. Knee exercises need to raise the patient's leg, keep the hip joint slightly bent, and then do knee flexion and extension activities. When training the ankle joint, bend the foot plate to the thumb and little toe in turn. Patiently instruct the patient to conduct balance training between sitting and standing positions. (4) Three to five weeks after admission: observe whether patients have joint limb reaction and joint movement and train their balance ability after the initial recovery of patients' motor ability. Patients were trained to walk on crutches as soon as they were able to stand. In walking training, patients can be first guided to alternate legs before and after the step, the center of gravity transfer, in the training of crutches first, out of the foot, and then keep up with the foot. After walking with crutches, you can practice walking on level ground, as well as up and down stairs and slopes. ⑤ 6 to 7 weeks after admission: assess patients' awareness of self-protection, observe their awareness and motor ability, and evaluate the effect of rehabilitation. ⑥ After leaving: the patient obtains the follow-up through phone calls once a week to understand the specific situation of the patient's limb recovery. At the same time, they were informed of the situation of taking medicine as prescribed and reminded to have regular check-ups in hospital. (2) Humanized nursing: ① psychological nursing: because cerebral infarction is more sudden onset, while causing damage to the physical function, it will also induce patients to produce anxiety, tension, fear, and other bad emotions, increasing the risk and instability of treatment. Therefore, it is necessary to timely assess the psychological status of patients, carry out targeted nursing according to the evaluation results to relieve or even eliminate the psychological pressure of patients, and increase the confidence in treatment. ② Environmental care: to create a good ward environment for patients, pay attention to ventilation, to ensure fresh air. At the same time, the temperature and humidity of the ward should be reasonably controlled. The temperature of the ward should be maintained at 19–24°C in summer and 18–20°C in winter, and the relative humidity should be controlled at 50%–60%. In addition, pay attention to ward health, towels, pillow towels, sheets, bedding, and other timely replacement. (3) Prevention of falling intervention: falling will not only yield a bad impact on patient's health and quality of life but also increase the difficulty of treatment. Therefore, fall prevention interventions are needed. First strengthen health education for patients and their families and increase their understanding of relevant matters needing attention. At the same time, carry out preventive skills education and training in order to helpfully prevent and respond to emergencies. Put the patient's daily articles in the place within their reach, easy for them to take, and then reduce the occurrence of falling bed, fall phenomenon. Strengthening night patrol is conducive to timely detection of patients' disease mutations and timely treatment to reduce the occurrence of adverse events. (4) Limb function nursing: massage the affected limb of the patient, according to the order of massage from far to near, and then effectively promote the circulation of local blood and lymph and eliminate swelling. When the patient's pain was considerably relieved, the affected area was massaged, and the patient was instructed to carry out the movement of wrist, elbow, toe, ankle, hip, knee, and other joints; the time was controlled at 15 min/time, twice a day Instruct the patient to slowly change from decubitus to sitting position, starting with 15° decubitus position and then increasing by 10°/day until increasing to 90°. Train the patient's walking ability by instructing him to extend his hips and then move his pelvis and torso horizontally. After the heel touches the ground, the knee maintains about 15° of flexion, then slowly straightens, but maintains flexion until the toe leaves the ground.

Both groups had been in nursing for 2 months.

### 2.4. Observation Indicators

① A comparison was made between the two groups about hospitalization expenses and days. ② Neurological function, daily living ability, and limb motor function: National Institute of Health Stroke Scale (NIHSS) [9], Barthel Index (Barthel Index), BI) [10], and Fugl-Meyer Motor Function Scale (Fugl-Meyer Assessment, FMA) [11], respectively, evaluated patients' neurological function, daily living ability, and limb motor function in both groups earlier than and after the nursing. The lower NIHSS score is, the higher BI and FMA score becomes and the better the body nerve function, daily living ability, and limb motor function are. ③ Complications and recurrence: pressure ulcers, urinary tract infection, stress ulcer bleeding, lung infection, and other complications and recurrence were observed in the two groups. (4) Satisfaction: the hospital satisfaction questionnaire was used to collect the evaluation of the two groups of patients on nursing. The evaluation grade is fairly satisfied, satisfied, and not satisfied: total satisfaction = fairly satisfied + satisfied.

### 2.5. Statistical Methods

SPSS 18.0 was employed to analyze statistics, and the measurement data were shown as mean ± standard deviation (±*S*). *T* was employed to make a test. Enumeration data were showed by example (*n*) or percentage (%) and examined by *χ*^2^. *P* < 0.05 pointed obvious difference in statistics.

## 3. Results

### 3.1. Comparison of Hospitalization Expenses and Days

The hospitalization expense and length of stay in the observation group were considerably lower than those in the control group, with obvious difference in statistics (*P* < 0.05), as shown in Table 2.

### 3.2. Comparison of Neurological Function, Daily Living Ability, and Limb Motor Function

There is no obvious difference in NIHSS, BI, and FMA marks between the two groups before nursing (*P* > 0.05). After nursing, NIHSS scores of the two groups were considerably decreased, while BI and FMA scores were considerably increased. NIHSS scores of the observation group were considerably lower than those of the control group, while BI and FMA scores were considerably higher than those of the control group, with obvious difference in statistics (*P* < 0.05), as shown in Table 3 and Figure 1.

### 3.3. Comparison of Complications and Recurrence between the Two Groups

The incidence and recurrence rate of complications in the observation group were considerably lower than those in the control group, and the differences were obvious in statistics (*P* < 0.05), as shown in Table 4.

### 3.4. Comparison of Nursing Satisfaction

The satisfaction with nursing in the observation group was considerably higher than that of the control group, and the distinction was obvious in statistics (*P* < 0.05), as shown in Table 5.

## 4. Discussion

Dyslipidemia, diabetes, heart disease, hypertension, etc., can promote the occurrence of cerebral infarction, mainly manifested as vertigo, consciousness disorder, ataxia, quadriplegia, etc., with high disability rate and fatality rate, which should be paid close attention to clinically [12]. At present, in addition to active and effective treatment for cerebral infarction patients, some nursing measures have been taken. However, clinical pathway nursing can provide comprehensive targeted nursing services for patients from aspects of illness, psychology, and so on [13]. The concept of humanized nursing service is to treat patients as nursing centers and provide them with high-quality and comprehensive care [14]. However, there are few research studies to make the application effect of clinical pathway nursing mixed with humanized nursing clear in cerebral infarction. The results of this study found that clinical pathway nursing combined with humanized nursing can usefully curtail the inpatient days, lower hospitalization expenditure, and improve neurological function, daily living ability, and limb motor function. Meanwhile, it can also lower the possibility of complications and recurrence rate and improve nursing satisfaction. The reasons are analyzed as follows.

Chen et al. [15] showed that NIHSS score of patients with cerebral infarction was considerably reduced after early pathway nursing. Fu et al. [16] showed that, after clinical nursing pathway was adopted for the intervention of patients suffering from acute intracerebral hemorrhage, the length of hospital stay was shortened and BI and FMA scores were considerably increased. In this study, the hospitalization cost and length of stay in the observation group were considerably less than those in the control group, and NIHSS scores in the two groups decreased after nursing, while BI and FMA scores increased. In contrast with the control group, the observation group had lower NIHSS scores and higher BI and FMA scores. Combined with the results of Chen and Fu, clinical pathway nursing combined with humanized nursing can effectively promote patient recovery, reduce hospitalization costs, and improve neurological function, daily living ability, and limb motor function. The reasons are analyzed. Its orientation is the nursing plan axis and the time axis. We optimize the clinical nursing process, clarify the specific nursing operation in each time period, implement targeted and planned nursing intervention, effectively identify and prevent emergencies in nursing, and then reduce the occurrence of emergencies. Moreover, it can actively guide patients to actively cooperate with the development of treatment and nursing and ultimately effectively shorten the recovery process of patients' physical health [17, 18]. Clinical pathway nursing was practiced in patients suffering from cerebral infarction; the first is to carry out health education for patients and promote the understanding of the disease and treatment of patients so that they actively cooperate with the development of treatment and nursing. After that, the patients were trained in language, body and other aspects, which promoted the recovery of patients. At the same time, it is conducive to the negative neurological function, which is conducive to improving patients' daily living ability and limb movement function. Humanized nursing, as a new nursing model, is developed from “humanized care.” Its core concept is people-oriented, starting from special requirements, thinking and interests, respecting patients' choice, providing them with optimal nursing services from various aspects, and promoting the development of nursing career [19, 20]. In this study, humanized nursing implemented psychological, environmental, fall prevention, limb function, and other aspects of the patient care; in the establishment of patient treatment confidence, we improve the treatment compliance at the same time, promote patient rehabilitation, and boost the patient's limb function. The combination of clinical pathway nursing and humanized nursing plays a synergistic part in promoting the rehabilitation of patients suffering from cerebral infarction and improving various functions of the body.

Li and Liu [21] showed that patients suffering from acute myocardial infarction who received the percutaneous coronary intervention were nursing after clinical pathway. Postoperative complications were considerably reduced and nursing satisfaction was considerably improved. In this study, the possibility of complications and the recurrence rate observation group was obviously lower than the control group, satisfaction with nursing is considerably higher than the control group, and Li's research results are basically consistent, suggesting that clinical pathway joint humanized nursing care used in patients with cerebral infarction can effectively decrease the complications and risk of recurrence and enhance patient satisfaction with care. Clinical path nursing is a targeted path table for disease treatment and follow-up care, which can not only effectively ensure the smooth implementation of treatment but also, in line with the specific condition of patients to adjust the nursing plan, effectively meet the needs of patients in all aspects. Meanwhile, the occurrence of complications can be diminished and the quality of nursing can be promoted [22, 23]. Humanized nursing respects patients' personal privacy, personality, and life value and is an effective, holistic, personalized, and creative nursing mode. It creates a comfortable treatment environment for patients and then makes patients feel satisfied, comfortable, and convenient [24, 25].

The limitation of this study is that the sample size is small, which may deviate the data results from the actual value. At the same time, long-term follow-up cannot be carried out, and the clinical path of combined humanized care cannot be determined. There will be a long-term impact of cerebral infarction, so it will take time to further expand the sample size and longer follow-up verification research.

## 5. Conclusion

In conclusion, clinical pathway nursing combined with humanized nursing in cerebral infarction can effectively reduce hospitalization costs, reduce the length of hospital stay, and improve neurological function, daily living ability, and limb motor function. Meanwhile, it can also reduce the risk of complications and recurrence and improve patient satisfaction with nursing care, which can be used as a reference for clinical research.

## Figures and Tables

**Figure 1:** Comparison of neurological function, activities of daily living, and limb motor function between the two groups before and after nursing. *Note.* In contrast with before nursing, ^*∗*^*P* < 0.05; in contrast with the control group, ^#^*P* < 0.05.

**Table 1:** Comparison of two groups of general data.

General data		Control group (*n* = 50)	Observation group (*n* = 50)	*t*/*χ*^2^ value	*P* value
Gender [*N* (%)]	Male	27 (54.00)	29 (58.00)	0.023	0.887
	Female	23 (46.00)	21 (42.00)		

Average age (years)		61.73 ± 9.63	61.14 ± 9.67	0.372	0.708

Mean time from onset to visit (h)		3.69 ± 0.26	3.50 ± 0.31	0.459	0.639

Severity of illness [*N* (%)]	Mild	22 (44.00)	23 (46.00)	0.473	0.492
	Moderate	15 (30.00)	16 (32.00)		
	Severe	13 (26.00)	11 (22.00)		

Infarct site [*N* (%)]	Basal ganglia area	17 (34.00)	18 (36.00)	0.454	0.501
	Lateral ventricle parabody	13 (26.00)	12 (24.00)		
	Thalamus	9 (18.00)	10 (20.00)		
	Bilateral frontal lobe	7 (14.00)	8 (16.00)		
	Temporal lobe area	4 (8.00)	2 (4.00)		

Education level [*N* (%)]	Junior high and below	26 (52.00)	25 (50.00)	1.516	0.681
	High school and technical secondary school	13 (26.00)	12 (24.00)		
	Junior college or above	11 (22.00)	13 (26.00)		

**Table 2:** Comparison of hospitalization expenses and length of stay between the two groups ($\bar{x}\pm s$).

Time	Control group (*n* = 50)	Observation group (*n* = 50)	*T* value	*P* value
Hospitalization expenses (YUAN)	14.73 ± 2.41	10.40 ± 1.34	5.189	0.022
Length of stay (days)	6978.30 ± 756.39	6438.53 ± 457.87	4.873	0.026

**Table 3:** Comparison of neurological function, activities of daily living, and limb motor function between the two groups before and after nursing ($\bar{x}\pm s$, score).

Project		Control group (*n* = 50)	Observation group (*n* = 50)
NIHSS score	Before the nursing	30.21 ± 3.25	29.86 ± 3.47
	After the nursing	17.63 ± 2.44^*∗*^	10.40 ± 2.23^*∗*#^
BI score	Before the nursing	42.30 ± 2.20	43.07 ± 1.54
	After the nursing	65.30 ± 5.23^*∗*^	85.33 ± 6.93^*∗*#^
FMA score	Before the nursing	52.30 ± 7.20	52.43 ± 7.03
	After the nursing	68.63 ± 8.20	86.74 ± 9.63^*∗*#^

Note: In contrast with before nursing, ^*∗*^*P* < 0.05; in contrast with the control group, ^#^*P* < 0.05.

**Table 4:** Comparison of complications and recurrence between the two groups [*n* (%)].

Project		Control group (*n* = 50)	Observation group (*n* = 50)	*χ* ^2^ value	*P* value
Complications	Pressure sores	5(10.00)	1(2.00)	—	—
	Urinary tract infection	5(10.00)	3(6.00)	—	—
	Stress ulcer bleeding	4(8.00)	3(6.00)	—	—
	Lung infection	8(16.00)	4(8.00)	—	—
Total		22(44.00)	11(22.00)	6.142	0.009
Recurrence		6(12.00)	1(2.00)	4.614	0.030

**Table 5:** Comparison of nursing satisfaction between two groups [*n* (%)].

Satisfaction	Control group (*n* = 50)	Observation group (*n* = 50)	*χ* ^2^ value	*P* value
Fairly satisfied	23(46.00)	34(68.00)	—	—
Satisfied	13(26.0)	14(30.00)	—	—
Not satisfied	14(28.00)	2(2.00)	—	—
Total	36(72.00)	48(96.00)	9.534	0.000

## Data Availability

The data used to support the findings of this study are available from the corresponding author upon request.
